# Role of GLI1 in Hypoxia-Driven Endometrial Stromal Cell Migration and Invasion in Endometriosis

**DOI:** 10.1155/2022/6890790

**Published:** 2022-10-15

**Authors:** Lili Wang, Jiaxin Liang, Siyi Bi, Yixuan Li, Wei Zhang, Wang Xiwen, Yi Liu, Hengwei Liu

**Affiliations:** ^1^Department of Obstetrics and Gynecology, Wuhan Fourth Hospital, Puai Hospital, Tongji Medical College, Huazhong University of Science and Technology, Wuhan, China; ^2^Department of Obstetrics and Gynecology, Union Hospital, Tongji Medical College, Huazhong University of Science and Technology, Wuhan 430022, China; ^3^Department of Obstetrics and Gynecology, Zhongnan Hospital of Wuhan University, Wuhan University, Wuhan 430071, China

## Abstract

Endometriosis (EMs) is a benign disease with the characteristics of invasion and migration, and its pathogenesis is related to hypoxia. The abnormal activation of glioma-associated oncogene homolog 1 (GLI1) plays an important role in the metastasis of multiple types of tumors. However, it is not clear whether GLI1 regulates the migration and invasion of endometrial stromal cells under hypoxic condition. Therefore, we use comprehensive analysis to explore the effects of hypoxic on GLI1 expression and their regulation on the pathogenesis of EMs. In this study, from immunohistochemistry, RT-qPCR, and western blot analysis, we discovered that the expression of hypoxia-induced factor-1*α* (HIF-1*α*) and GLI1 was significantly increased in eutopic and ectopic endometrium of patients with EMs. In human primary eutopic endometrial stromal cells (ESCs), hypoxia can increase the expression of HIF-1*α* and GLI1 in a time-dependent manner. And hypoxia could promote GLI1 expression in a HIF-1*α*-dependent manner. Moreover, data from transwell assays manifested that the migration and invasion ability of ESCs was significantly enhanced under hypoxia, and this effect could be reversed by silencing GLI1. Furthermore, the expression of MMP2 and MMP9 was also increased under hypoxia, while silencing GLI1 could reverse this event. In summary, our research verified that GLI1, which activated by hypoxia, may contribute to the migration and invasion of ESCs through the upregulation of MMP2 and MMP9 and can be a novel therapeutic target in EMs.

## 1. Introduction

Endometriosis (EMs) is defined as the presence of endometrial tissue (glandular epithelium or stromal cells) outside the uterine cavity, concurrent adhesion, invasion, and growth. According to statistics, EMs affect 6% to 10% of reproductive-age women. It is the main cause of pelvic pain and infertility in women of productive age and seriously interferes with women's reproductive health [1, 2]. Numerous theories have been put forward for the pathogenesis of EMs, including retrograde menstruation, coelomic metaplasia, lymphatic and venous dissemination theory, and immune defense deficiency theory [3]. The most widely accepted theory, retrograde menstruation theory, refers to endometrial fragments retrograde into the pelvis through the fallopian tube during the menstrual cycle, then implant in the abdominal organs, resulting in chronic inflammation and adhesion [4, 5]. However, there are still defects in this explanation, and so far, there is no one theory that can fully explain the pathogenesis of EMs.

Hypoxia is not only a critical factor involved in a variety of pathophysiological processes but also an important microenvironment for the pathogenesis of EMs [6, 7]. According to retrograde menstruation theory, the blood supply was lost, and the hypoxia environment appeared after the endometrium fell off. Retrograded endometrial fragments in the pelvic may undergo certain changes under this microenvironment to combat the scarcity of nutrients and the accumulation of stress. Studies have shown that pelvic hypoxia could affect the occurrence and development of EMs by regulating the synthesis and response of estrogen [8, 9], angiogenesis [10], and epigenetic [11].

The Hedgehog signaling pathway is highly conserved in the process of biological evolution, while glioma-associated oncogene 1 (GLI1) is the core downstream transcription factor of this signaling pathway [12]. Abnormal activation of GLI1 leads to increased transcription of target genes, which regulates a variety of cellular biological processes, including proliferation, apoptosis, migration, and invasion [13–15]. At present, higher expression of the GLI1 gene has been observed in multiple malignant tumors, including hepatocellular carcinoma [16] and pancreatic cancer [17]. It plays an important role in tumor invasion and metastasis. Although EMs are regarded as a benign disease, ectopic endometrial cells show malignant biological characteristics and have a stronger ability of invasion, migration, and abnormal proliferation compared with normal types [18]. Previous study [19] has demonstrated that GLI1 was elevated in eutopic endometrium of EMs; however, whether GLI1 may play a critical role under hypoxic environments in the development of EMs is still poorly understood.

In the present study, we aimed to clarify the relationship between the GLI1 gene and the pathogenesis of EMs and also to determine the role of GLI1 in the invasion of EMs mediated by hypoxia. This study provides novel theoretical basis and treatment strategy for the pathogenesis of EMs.

## 2. Materials and Methods

### 2.1. Patients and Tissue Collection

The patients were recruited from the Department of Obstetrics and Gynecology, Union Hospital, Tongji Medical College, Huazhong University of Science and Technology between June 2017 and October 2018. The normal endometrial tissues of 30 healthy women with infertility due to male factors, ectopic endometrium tissues, and corresponding eutopic endometrial tissues of 30 patients with ovarian endometriosis were collected. According to the standard of the American Society of Reproductive Medicine (ASRM), it is classified as stage I-IV EMs [20]. The ectopic endometrial tissue was separated by laparoscopy, and the corresponding eutopic endometrial tissue was separated by hysteroscopy. All specimens were collected during the proliferative phase of the normal menstrual cycle. The tissue samples were collected using the Nowak's curette just before the surgical procedure, and transported to the laboratory for research use. This study was approved by the Ethics Committee of Tongji Medical College of Huazhong University of Science and Technology (IORG No: IORG0003571), and all the above patients signed informed consent. All fresh specimens were frozen and stored in liquid nitrogen to further extract protein and RNA. The clinical data about the patients are reported in Supplemental Table 1.

### 2.2. Human Primary Eutopic Endometrial Stromal Cells (ESCs) Isolation and Cell Culture Conditions

Isolation of primary eutopic endometrial stromal cells from eutopic endometrium of infertile patients with EMs. The collected fresh tissue was placed on ice, washed with precooled PBS, and shredded to 1 mm^3^ size tissue homogenate. Type II collagenase (0.1%, Sigma Aldrich, MO, USA) was added to digest for 60 min at 37°C. The tissue homogenate was filtered through aseptic 400 *μ*m and 100 *μ*m sieves, respectively, to remove undigested tissue and epithelial cells. The supernatant was discarded after 1000 rpm/min centrifugation for 5 min. Then the red blood cell lysate reagent (Beyotime, Shanghai, China) was added and mixed well to make it fully cleaved. After 1000 rpm/min centrifugation for 5 min, supernatant was discarded and cells were suspended with 2 ml DMEM/F12 medium containing 10%FBS (Gibco, CA, USA) and cultured at 37°C.

### 2.3. Immunohistochemistry Staining

The paraffin-embedded fresh tissue specimen was stained by immunohistochemical staining according to the standard procedure. Soak the sample in 3% hydrogen peroxide solution at room temperature and incubate with the primary antibody overnight at 4°C. The secondary antibody labeled with biotin was incubated at room temperature for 2 hours and washed with PBS 3 times, incubated with diaminobenzidine (DAB) and hematoxylin, and observed and photographed under the microscope. The primary antibody used included the following: anti-HIF1*α* (Affinity, AF1009, 1 : 100) and anti-GLI1 (Abcam, ab217326, 1 : 100). The immunostaining score of HIF-1*α* and GLI1 protein in endometrial tissues is presented in Supplemental Table 4.

### 2.4. RNA Extraction and Quantitative Real-Time Polymerase Chain Reaction (qRT-PCR)

The qRT-PCR assay was performed according to our previous study [21]. The total RNA of ESCs was collected by TRIzol reagent (Vazyme Biotech, Nanjing, China), and the RNA was reverse transcribed into cDNA by HiScrip II QRT SuperMix (Vazyme Biotech, Nanjing, China). The expression level of mRNA was calculated by the method of 2^−*ΔΔ*Ct^. The primer sequences used for real-time RT-PCR are presented in in Supplemental Table 2.

### 2.5. Western Blot

The total proteins of ESCs were collected by radioimmunoprecipitation assay buffer (RIPA) (Beyotime Biotechnology, China) and quantified by bicinchoninic acid assays (Beyotime, Shanghai, China). The protein samples were denatured after incubation at 95°C for 10 minutes. Target proteins were separated by 12% SDS-PAGE and transferred to a polyvinylidene fluoride membrane, sealed with 5% skim milk at room temperature for 1 hour, incubated overnight with the primary antibody, and then soaked with the secondary antibody. The primary antibody used included the following: anti-HIF-1*α* (Affinity, AF1009, 1 : 1000), anti-GLI1 (Abcam, ab217326, 1 : 1000), anti-MMP2 (Affinity, AF5330, 1 : 1000), anti-MMP9 (Affinity, AF5228, 1 : 1000), anti-GAPDH (ProteinTech, 10494-1-AP, 1 : 20000). The commercial sources and characteristics of antibodies used are summarized in Supplemental Table 3.

### 2.6. Cell Transfection

For adenoviral transduction, ESCs in the logarithmic phase were digested and inoculated on a 6-well plate according to 5 × 10^4^/ml. When the cell density reached 50-60%, the cells were ready to be transfected. Before infection, the medium was replaced by 1 ml fresh complete medium. The control shRNA adenovirus vector and GLI1 shRNA adenovirus vector (multiplicity of infection (MOI) = 50) were added, respectively. After cultured for 24 hours, fresh complete medium was replaced to continue the culture for another 24 hours, and the fluorescence expression of GFP was detected under the fluorescence (IX51, Olympus, Tokyo, Japan) inverted microscope. If the fluorescence rate in the visual field was more than 80%, the follow-up experiment could be carried out.

For siRNA transient transfection, 50 nmol/l siRNA-HIF-1*α* was transfected into ESCs by using Lipofectamine 2000 Reagent (Thermo Scientific, Waltham, MA, USA) and OPTI-MEM (Invitrogen, USA) according to the manufacturer's protocol. All the RNA oligoribonucleotides were purchased from RiboBio (RiboBio, Guangzhou, China). The primer sequences used for siRNA analyses are presented in in Supplemental Table 2.

### 2.7. Transwell Migration and Invasion Assays

The migration and invasive ability of ESCs was evaluated by transwell assay. For invasion assay, the superior chamber was precoated with 50 *μ*l of Matrigel (2 mg/ml) (Becton, Dickinson and Company) and incubated at 37°C for at least 4 h. Then cells were resuspended with serum-free DMEM/F12 medium after digestion, and the cell concentration was adjusted to 1 × 10^6^ cells/ml after counting. The 200 *μ*l cell suspension was added to the upper surface of the chambers. 500 *μ*l complete medium containing 10% FBS was added into the lower chamber. After being incubated at 37°C for 24 hours, the chamber was taken out. The chamber was cleaned with PBS, fixed with paraformaldehyde and stained with 0.1% crystal violet, and observed under the microscope (Nikon Eclipse TE2000U inverted microscope with a CCD camera).

### 2.8. Statistical Analysis

The experimental results in this study were repeated three times independently, and the GraphPad Prism8.0 software was used to analyze. The data that passed normality test were determined by applying Student's *t* test and one-way analysis of variance followed by Tukey's post hoc test among more than two groups. For all statistical tests, *P* < 0.05 was considered significant.

## 3. Results

### 3.1. Expressions of GLI1 and HIF-1*α* in Ovarian Endometriosis

Immunohistochemical was used to determine the expression of HIF-1*α* and GLI1 in normal endometrium and eutopic and ectopic endometrium of EMs. The results showed that HIF-1*α* was located in both the cytoplasm and nucleus of glandular epithelial cells and stromal cells in endometrial tissue. Compared with normal endometrium, the expression of HIF-1*α* in ectopic endometrium was remarkably increased, but there was no significant difference in eutopic endometrium (Figure 1(a) (A–F)). Strong GLI1 expression was observed in the cytoplasm of glandular epithelial cells in normal endometrium, while it is mainly located in the nucleus in eutopic and ectopic endometrium of EMs (Figure 1(a) (G–I)). Besides, it was also observed that a significant increase in the expression of GLI1 in eutopic and ectopic endometrium of patients with EMs when compared with normal endometrium (Figure 1(a) (G–I)). To further compare the expression of GLI1 and HIF-1*α* in ovarian endometriosis, qRT-PCR and western blot assays were also performed. The results showed that the mRNA and protein expression of GLI1 in eutopic and ectopic endometrium of patients with EMs was significantly higher than those in normal proliferative endometrium (Figures 1(b)–1(d)). As for HIF-1*α*, the expression level of mRNA and protein was also significantly increased in ectopic tissues, but no significant change was observed between eutopic and normal endometrium (Figures 1(b)–1(d)). These results indicated that these two genes may both play an important role in the development of EMs. However, whether there was a connection between HIF-1*α* and GLI1 remained unknown.

### 3.2. Hypoxia Promotes GLI1 Expression of the ESCs in a HIF-1*α*-Dependent Manner

To clarify whether the expression of GLI1 and HIF-1*α* was associated with hypoxia, we performed qRT-PCR and western blot assays for isolated eutopic endometrial stromal cells (ESCs) under hypoxia treatment. As shown in Figures 2(a)–2(c), RT-PCR and western blot results indicated that a time-dependent increase in both HIF-1*α* and GLI1 mRNA and protein expression were observed. Furthermore, we also knockdown the expression of HIF-1*α* by specific siRNA under hypoxia condition to investigate the role of HIF-1*α* in hypoxia induced GLI1 activation. The results suggested that compared with ESCs cultured under hypoxia condition, decreased expression of HIF-1*α* and Beclin1 and GLI1 was observed in ESCs transfected with HIF-1*α* siRNA under hypoxia condition (Figures 2(d)–2(f)). These suggest that GLI1 activation under hypoxic condition was dependent on the status of HIF-1*α*.

### 3.3. Hypoxia Promotes Invasion of Endometrial Stromal Cells in a GLI1-Dependent Manner

To investigate the biological function of GLI1 under hypoxia condition, we constructed an empty adenovirus and GLI1 shRNA recombinant adenovirus vectors. Transwell migration and invasion assays showed that the invasive ability of cells was significantly enhanced under hypoxia when compared with the normoxic group, while silencing the GLI1 gene can effectively reverse this effect (Figures 3(a)–3(d)). These evidences indicated that the enhanced invasion of eutopic endometrial stromal cells in EMs mediated by hypoxia was depended on GLI1 expression.

### 3.4. GLI1 Contributed to EMs Invasion through Upregulation of MMP2 and MMP9

Given the importance of matrix metalloproteinases family genes (MMPs) in the process of cell migration and invasion, we focused on the effects of GLI1 on the expression of MMP2 and MMP9 under hypoxia. It was shown that the mRNA and protein expression of GLI1, MMP2, and MMP9 was markedly higher under hypoxia when compared with normoxia (Figures 4(a)–4(c)). To further determine its internal relationship, we silenced GLI1 under hypoxia and sought to clarify whether the upregulation of MMP2 and MMP9 under hypoxia could be attributed to GLI1. The results of qRT-PCR and western blot assays showed that both MMP2 and MMP9 diminished after GLI1 silencing under hypoxic conditions (Figures 4(a)–4(c)). Collectively, the findings suggested that the ability of GLI1 to promote invasion under hypoxia may be realized by MMP2 and MMP9.

## 4. Discussion

Endometriosis is an estrogen-dependent chronic gynecological disease. The pelvic pain, infertility, and increase in the risk of epithelial ovarian cancer caused by EMs triggered a serious physical, mental, and financial burden on women. Up to now, there is still no typical conclusion on the specific pathogenesis of EMs [22]. The lack of detailed knowledge about this disorder also leads to barren and ineffective treatments. Despite receiving drug or surgical treatment, EMs patients still face a high risk of recurrence and long-term drug side effects [23]. Therefore, it is of great clinical significance to explore the molecular mechanism of the occurrence and development of endometriosis and to find specific sites to achieve the targeted therapy of EMs.

Hypoxia is a usual phenomenon, and it is one of the most common features in the solid tumor microenvironment. Hypoxia has been widely reported to be related to the invasive phenotype of tumors, including cell proliferation, angiogenesis, and drug resistance, [24–28]. Extensive studies have confirmed that the effect of hypoxia on tumor invasion is achieved through the transcriptional activation of different genes by hypoxia-induced factor [29–31]. Although it is not a tumor, EMs also shows many malignant features similar to tumors, such as strong invasion and migration [18, 32, 33]. In this study, we found that the expression of HIF-1*α* was increased in ectopic lesions of patients with EMs. After continuous hypoxia stimulation of eutopic endometrial stromal cells, HIF-1*α* elevated in a time-dependent manner. Hypoxia-induced factor-1*α* (HIF-1*α*) is the main factor in cell response to hypoxia stress. Under hypoxia conditions, HIF-1*α* forms dimer with HIF-1*β* and together regulates downstream by interaction with hypoxia response element (HRE) [34]. The augment expression of HIF-1*α* in ectopic lesions suggests that hypoxia plays an essential role in the occurrence and development of EMs.

Similarly, besides HIF-1*α*, we found that the expression of GLI1 increased in ectopic lesions and also showed upregulated expression in a time-dependent manner to hypoxia. Moreover, hypoxia could upregulate GLI1 through HIF-1*α* activation. GLI1 is at the terminal end of the highly conserved Hedgehog signaling (Hh) pathway. When GLI1 is released, it can trans into the nucleus to regulate gene transcription as a transcription factor [35]. Abnormal activation of the Hh pathway can lead to various biological events such as cancer stem cell self-renewal, growth, invasion, and migration [36–39]. As the terminal molecule of the Hh signaling pathway, the occurrence of these malignant events is closely related to GLI1. Therefore, we speculate that the high expression of GLI1 in patients with EMs may be the culprit of downstream malignant events. We found that the enhancement of hypoxia-induced migration and invasion abilities in eutopic endometrial stromal cells was attenuated after silencing of GLI1 gene. These findings prove that the highly expressed GLI1 can contribute to hypoxia-induced invasion enhancement in EMs.

As a transcription factor, GLI1 functions mainly by regulating the expression of downstream genes. We speculate that GLI1 may affect cell migration and invasion by regulating matrix metallopeptidases (MMPs). MMPs have been found to degrade extracellular matrix and basement membrane [40]. It is frequently found in malignant tumors and is closely related to invasion and migration [41–43]. Li et al. [44] found that programmed cell death 4 (PDCD4) can attenuate the expression of THE NF-*κ*B/MMP2/MMP9 signaling pathway, thus attenuating the migration and invasion potentiality of human endometrial stromal cells. This suggests that MMPs may play a role in the migration and invasion of EMs. It was found that the expression of MMP2 and MMP9 was significantly augmented under hypoxia, and this event could be reversed by silencing of GLI1. This indicates that GLI1 could regulate migration and invasion of endometrial stromal cell through MMP2 and MMP9.

However, our current study has some limitations. Firstly, only proliferative phase endometrium was analyzed, and the sample size was relatively small, which may reduce the interpretable power of the data. Therefore, large sample size from an entire menstrual cycle should be studied in our future research. Second, the exact molecular regulatory mechanisms underlying GLI1 mediated MMP2/9 upregulation in human endometrial stromal cells remains to be elucidated. Last but not least, only late-stage ovarian endometriosis sample was used, and the results may provide little insight into peritoneal and deep infiltrating lesions. Therefore, future research is needed to pay more attention into these questions.

In conclusion, we have first uncovered a novel link between hypoxia microenvironment and GLI1 in the pathogenesis of endometriosis. Our results presented that GLI1 has a significant higher expression in ovarian endometriosis and is correlated with elevated expression of HIF-1*α*. We further demonstrate that hypoxia can induce the expression of GLI1 in ECS cell, which then promotes cell migration and invasion through the MMP2/9 pathway (Figure 5). Overall, the HIF1*α*-GLI1-MMPs axis will be a potential therapeutic in ovarian endometriosis.

## Figures and Tables

**Figure 1:** Differential expression of GLI1 and HIF-1*α* in normal, eutopic and ectopic endometrial tissues. (a) Immunohistochemistry assay was performed to confirm the expression and localization of HIF-1*α* and GLI1 protein in normal proliferative endometrium (A, B, G, and H), eutopic endometrium (C, D, I, and J), and ectopic endometrium (E, F, K, and L). The images were observed under 200 times and 400 times visual field. (b) The relative expression levels of GLI1 and HIF-1*α* in eutopic (*n* = 40) and ectopic (*n* = 40) endometrial specimens from patients with ovarian endometriosis (EMs) and normal endometrial (*n* = 40) specimens were measured by (b) qRT-PCR and (c, d) western blot. Statistical analysis was conducted by the Kruskal–Wallis test. The data are presented as the mean ± SD of three independent experiments. ^∗^*P* < 0.05, ^∗∗^*P* < 0.005 by one-way ANOVA.

**Figure 2:** Hypoxia promotes GLI1 expression of the ESCs in a HIF-1*α*-dependent manner. (a) GLI1 and HIF-1*α* expression in ESCs was detected by qRT-PCR following treatment with hypoxia at a series of time points (0, 8, 16, 24, and 48 hours). (b, c) GLI1 and HIF-1*α* protein expression in ESCs was determined following treatment with hypoxia at indicated time points (0, 8, 16, 24, and 48 hours). (d–f) ESCs were transfected with HIF-1*α*-specific siRNA in the presence of hypoxia, and then the expression of GLI1 and HIF-1*α* mRNA and protein was measured by qRT-PCR and western blot. The data are presented as the mean ± SD of three independent experiments. ^∗^*P* < 0.05, ^∗∗^*P* < 0.005 by one-way ANOVA.

**Figure 3:** Inhibition of GLI1 attenuates the migration and invasion capacities of ESCs. (a, b) Transwell assays showed the migration capacities of ESCs infected with scramble shRNA and GLI1 shRNA. (c, d) Transwell assays showed the invasion capacities of ESCs infected with scramble shRNA and GLI1 shRNA. All images were taken at ×200 magnification. The data are presented as the mean ± SD of three independent experiments. ^∗^*P* < 0.05, ^∗∗^*P* < 0.005, ^∗∗∗^*P* < 0.001 by one-way ANOVA.

**Figure 4:** GLI1 contributed to EMs invasion through upregulation of MMP2 and MMP9. (a, b) GLI1, MMP2, and MMP9 mRNA and protein expression was determined by qRT-PCR and western blot in ESCs treated with normoxia, hypoxia, hypoxia + scramble shRNA, and hypoxia + GLI1 shRNA. The data are presented as the mean ± SD of three independent experiments. ^∗^*P* < 0.05, ^∗∗^*P* < 0.005, ^∗∗∗^*P* < 0.001 by one-way ANOVA.

**Figure 5:** A brief schematic diagram depicting how hypoxia promote migration and invasion by regulating GLI1 mediated MMP2 and MMP9 expression in human eutopic endometrial stromal cells (ESCs).

## Data Availability

The datasets generated during and/or analyzed during this study are available from the corresponding author on reasonable request.

## Supplementary Materials

Supplementary Materials Table S1: clinical characteristics of patients. Table S2: primer sequences used for real-time RT-PCR and siRNA analyse. Table S3: commercial sources and characteristics of antibodies used. Table S4: immunostaining score of HIF-1*α* and GLI1 protein in normal endometrium, eutopic endometrium and ectopic endometrium of endometriosis.
